# Risks of Misinterpretation in the Evaluation of the Effect of Fruit-Based Drinks in Postprandial Studies

**DOI:** 10.1155/2014/870547

**Published:** 2014-12-25

**Authors:** Ilaria Peluso, Maura Palmery

**Affiliations:** ^1^Food and Nutrition Center of the Agricultural Research Council (CRA-NUT), Via Ardeatina 546, 00178 Rome, Italy; ^2^Department of Physiology and Pharmacology “V. Erspamer”, “Sapienza” University of Rome, Piazzale Aldo Moro 5, 00185 Rome, Italy

## Abstract

It has been suggested that some fruit-based drinks (FBD) may delay the onset of postprandial stress, which is involved in the pathogenesis of many diseases. The majority of the studies, which have investigated the effects of FBD on postprandial stress, involved a placebo that was a drink with the same content in sugars or carbohydrates of the FBD, but without the bioactive antioxidant compounds. These studies were aimed more at evaluating the effect of the antioxidants rather than the effect of the FBD as a whole. Only 4 studies compared the effect of FBD with water as control and did not support the hypothesis that FBD could inhibit postprandial dysmetabolism, as well as the studies that compared the effect of orange juice and cola. Overall, the results suggest a complex relationship between postprandial dysmetabolism, inflammation, and oxidative stress. Furthermore, the inflammatory and oxidative stress markers need further analytical validation and normal ranges should be established in order to reach a firm conclusion. Finally, caution should be taken in the interpretation of the effect of FBD in postprandial studies and the reviewed results suggest that dietary recommendations should aim to limit rather than increase sugar-sweetened beverages consumption.

## 1. Introduction

The frequent consumption of high fat (HFM), high carbohydrates (HCM), or mixed high fat and high carbohydrates (HFHCM) meals is associated with an increased risk of diabetes and cardiovascular disease (CVD) [1–3]. This association seems attributable to the onset of a condition defined as “low-grade chronic inflammation,” which is mediated by inflammatory cytokines and oxidative stress [4]. In particular, some cells associated with the innate immune response respond to the acute postprandial lipid increase with the oxidative burst [4]. It has been suggested that some fruit-based drinks (FBD) may delay the onset of postprandial stress [2, 3].

However, although FBD contain many flavonoids that act as antioxidants [3, 5], the human studies, which have investigated the effect of these polyphenols on immune function, have given contrasting results [3, 6]. Moreover, it has been suggested to avoid soft drinks containing sugars, including fruit juices that contain a lot of fructose, in the nutritional management of nonalcoholic fatty liver disease (NAFLD) [7], inflammatory bowel disease (IBD), and irritable bowel syndrome (IBS) [8].

We aim to review the results of the studies that have investigated the effects of FBD by using the postprandial stress as acute model of inflammation, taking into account the control used for the comparison.

## 2. The Postprandial Stress as Acute Model of Inflammation

It has been suggested that the dynamic models of acute inflammation may provide much more sensitive and meaningful information of the health state of an individual, with respect to the assessment of fasting inflammatory and metabolic markers [1]. The models of acute inflammation can be classified on the basis of the dominant event that triggers the inflammatory response and may therefore be divided into metabolic overload (oral glucose or lipids), stress from infection (injection of the endotoxin lipopolysaccharide, LPS), hypersensitivity responses to vaccines, and tissue damage (strenuous exercise or exposure to UV light) [1].

In Western society, the two prevalent origins of oxidative stress are the ingestion of HFM and the performance of strenuous exercise. However, in exercise-trained men, the magnitude of oxidative stress following HFM is significantly greater than that elicited by either aerobic or anaerobic exercise [24]. On the other hand, exercise improves postprandial glucose metabolism [25, 26] and the activation of leukocytes induced by lipaemia [27, 28]. However, exercise does not influence postprandial triglycerides (TG) and oxidative stress in obese prediabetic women [29]. In fact, obesity and type 2 diabetes (T2D) are considered important factors in the extent of postprandial stress, which is greater in subjects with the metabolic syndrome [1]. The extent of the postprandial inflammatory response seems to be correlated with the degree of insulin resistance [30, 31]. We have recently suggested that repeated hyperinsulinemia could be induced to inhibit the postprandial inflammation [4]. On the other hand, the increased activation of leukocyte in T2D may be due to the fact that metabolic diseases and obesity are associated with an increased intestinal permeability and an increased translocation of LPS from the lumen to the mucosa [1, 4, 32]. In fact, the most accepted mechanism of the postprandial activation of leukocyte is the phenomenon known as metabolic endotoxemia [4, 32]. The endotoxemia may be caused by direct spread of the LPS from the intestinal lumen, due to increased intestinal paracellular permeability, or through the absorption by enterocytes during the process of secretion of chylomicrons [4, 32]. HFHCM induces an increase of LPS and inflammatory cytokines [4]. The primary role of lipids, in the postprandial endotoxemia, is supported by the evidence that while HFM increased the levels of tumor necrosis factor-alpha (TNF-*α*), interleukin 1-beta (IL-1*β*), LPS, and Toll-like receptor-4 (TLR4), the ingestion of glucose increased only TNF-*α* and IL-1*β* [33]. TLR4, along with the LPS receptor (CD14), is involved in the induction of the oxidative burst and may be involved also in the activation of monocytes by urate crystals that form in the case of hyperuricemia [4]. Therefore, the increase in uric acid (UA) after HFM could enhance the innate immune response and the production of reactive oxygen species (ROS) [4]. In this context, it has been suggested that dietary fructose may increase plasma UA [34] and it is well known that fructose overfeeding increases fasting and postprandial plasma TG concentrations, which are related to the stimulation of hepatic de novo lipogenesis and to a decreased clearance of TG-rich lipoproteins [35–39]. The dyslipidaemic effect of dietary fructose occurs also in healthy children and is higher in those with NAFLD [40]. On the contrary, it has been recently reported that moderate amounts of high fructose or high glucose sweetened beverages for 2 weeks did not have differential effects on postprandial TG in physically active adolescents [41]. These results could be due to the lowering effect of exercise on the percentage of CD14 positive cells, the TLR4 expression, the LPS-stimulated production of TNF-*α*, and the increases in ROS, all induced by postprandial lipaemia [27, 28]. The role of CD14, TLR4, LPS, and TNF-*α* in the development of NAFLD [42–44] could account also for the protective effect of the physical activity in this disease.

## 3. The Effect of FBD on Postprandial Stress

Some studies have investigated the effects of FBD on postprandial stress (Tables 1 and 2) [9–23].

The postprandial glucose increase is characterized by a peak at around 30 minutes after the meal; then, glucose returns to baseline approximately two hours after the meal (in healthy subjects), consistent with the insulin response. On the other hand, the majority of the studies that evaluated the effect of HFM recorded a peak of TG 3–5 hours after the meal. Increases in inflammatory cytokines can be found with a peak between 3 and 6 hours after the meal and TNF-*α* in particular has a significant role in the oxidative burst induced by postprandial lipaemia [4]. Therefore, in order to follow the inflammatory response, markers of inflammation and oxidative stress were analyzed, in particular, the cytokines, the oxidative burst, the products of lipoperoxidation, and the nonenzymatic antioxidant capacity (NEAC) (Tables 1 and 2).

In the studies reported in the literature (Tables 1 and 2), the quality and the quantity of the ingested fats vary widely and often the effect of the simultaneous consumption of sugars and lipids was analyzed. The majority of the studies involved a placebo that was a drink with the same sugars or carbohydrates (CHO) content of the FBD, but without the bioactive antioxidant compounds (polyphenols and vitamin C). These studies were aimed more at evaluating the effect of antioxidants rather than the effect of FBD as a whole (Table 1) [9–19]. Furthermore, Snyder et al. [19] aimed to evaluate the effect of polyphenols contained in navel orange juice; therefore, they used a placebo matched in energy, sucrose, fructose, glucose, and ascorbic acid (Table 1). On the other hand, only 4 studies evaluated the effect of FBD with water as control (Table 2) [20–23].

### 3.1. Studies with Placebo Matched in Carbohydrates

Eleven studies (14 interventions) [9–19] investigated the effect of FBD by using a placebo matched in CHO (Table 1). Only in two interventions [9, 11] the subjects received a HFM with the placebo beverage at the end of a period of 6 weeks of supplementation with either a strawberry or a placebo beverage. The same HFM, HCM, or HFHCM was used in each study and sometimes the same meal was used in different studies (Table 1). Three studies [9–11] used a test meal composed of bagel (110 g), cream cheese (14 g), margarine (5 g), hard-boiled egg (50 g), and whole milk (240 g). Three studies [16–18] used a meal composed of fried potatoes (212 g), fried eggs (108 g), cheese (90 g), and white bread (90 g). Two studies [13, 15] used a meal consisting of one EggMcMuffin, one Sausage McMuffin, and two hash brown patties. The other three studies used 200 g of cream and 75 g of sucrose [12], high-oleic sunflower oil baked into a muffin [14], or 28 g of Kellogg's Corn Flakes and 118 mL of 2% milk [19].

The majority of the interventions did not affect postprandial TG (55.5%), total cholesterol (TC, 75%), insulin (80%), and glucose (87.5%). Only 3 interventions reported decreased levels of TG in overweight (OW) subjects, of which two involved dyslipidaemic individuals [9] and one involved a meal containing 81 g of fat and a FBD containing not only fruit juices and extracts (Table 1) but also a tea extract [18]. In this context, it is known that tea catechins reduce TG absorption [45] and that 80 g of lipids induced a marked effect on postprandial TG [3]. On the other hand, Mathew et al. [14] observed different effects on TG and glucose when the FBD was consumed during (DUR) or 15 min before (PRE) the HFM. The drink contained a pomegranate extract and caused a greater increase in postprandial TG after PRE compared to control, whereas a mean increase of 0.44 mmol/L in plasma glucose concentrations was found following DUR compared to the mean decreases of −0.25 mmol/L and −0.26 mmol/L following control and PRE, respectively.

Only Edirisinghe et al. [10] reported that postprandial plasma insulin concentrations in OW dyslipidaemic individuals were significantly lower, compared to the placebo beverage, when a strawberry beverage was consumed with the test meal. However, plasma glucose concentrations were not different between the treatments. Furthermore, the placebo used in the studies of this group [9–11] was matched in sugars (51.6) but had a different content of white granulated sugar (10 g) compared to the strawberry beverage (3 g).

Kay and Holub [13] reported that serum glucose concentrations were significantly higher in the blueberry group at 3 and 4 h than in control, in accordance with the delayed onset of postprandial glucose after fructose ingestion [46].

In dyslipidaemic subjects, the postprandial TG levels were significantly lower, compared with placebo, when a strawberry beverage was consumed with HFM or for 6 weeks before the test meal plus placebo [9]. The strawberry beverage decreased the oxidized low density lipoproteins (oxLDL) both when it was consumed with the HFM and when it was consumed for 6 weeks before the HFM challenge. On the other hand, the decrease in IL-6 was observed only when strawberry beverage was consumed during the HFM and no effect was observed on TNF-*α* and IL-1*β* (Table 1).

Concerning the effect of FBD on the postprandial increase of cytokines, TNF-*α* and IL-6 decreased, respectively, in 40% and 60% of the interventions (Table 1).

On the contrary, Huebbe et al. [12] in OW atherosclerosis-prone phenotype subjects, using a FBD and a placebo beverage identical in energy, sucrose, fructose, and glucose, adjusted for dietary fibre content and different in ascorbic acid (122 mg/250 g) and total polyphenol content (617 mg gallic acid equivalents/250 g), observed an increase in the postprandial IL-6 (plasma values) and TNF-*α* (*ex vivo*), despite the increase of NEAC and ascorbic acid and the nonsignificant effect on IL-1*β* (*ex vivo*), oxLDL, glucose, insulin, TG, and TC.

The lipoperoxidation markers decreased in 50% of the interventions, whereas an increase in NEAC was observed in 83.3% of the interventions. Despite the fact that the consumption of HFHCM has been associated with oxidative stress and with a decline in antioxidant defences in plasma, increases in NEAC have been reported following HFM [13, 16]. The increase in TG over time, but not serum glucose, was positively correlated with the increase in NEAC [13]. In OW subjects, after the consumption of a HFM, increased UA levels were documented, in conjunction with an increase of TG, TNF-*α*, and IL-6 [47]. The increase in endogenous antioxidants after HFM could account for the increase of NEAC [47]. Despite the ability of fructose to increase UA, two FBD with a different antioxidant capacity and with a different fructose content (FBD1: total radical-trapping antioxidant parameter (TRAP) 16.4 mM, ferric reducing antioxidant potential (FRAP) 27.6 mM, and fructose 57 g/L; FBD2: TRAP 9.7 mM, FRAP 13.6 mM, and fructose 29 g/L)) showed the same inhibitory effect on UA, which reached a peak 2 h after HFM [16]. On the other hand, only the FBD1 intervention significantly increased the urinary and plasma NEAC.

Overall, the studies that have investigated the effect of the antioxidants contained in FBD on postprandial stress (Table 1) have given contrasting results due to the differences in fat and CHO content of the meal and in glucose and fructose content of the placebo beverage.

### 3.2. Studies That Evaluated the Effect of Fruit Juice

Studies that evaluated the effects of fruit juices on HFM or mixed meals with water as control in healthy subjects are described in Table 2. Two of these studies compared also the effect of orange juice and drinks matched in sugars (placebo or cola) on postprandial glucose. Total calories from the intake of beverage with pizza were higher following the caloric beverages (orange juice and regular cola) compared to either water or diet cola [22]. Authors found higher blood glucose after the meals with orange juice and regular cola compared to diet cola and water [22]. Also Sullivan and Scott [48], in non-insulin-dependent diabetes mellitus patients, found no difference in the postprandial serum glucose after Coke or orange juice consumption. Cola and orange juice were the beverages of the two isocaloric meals (820 kcal, 41% fat, and 42% CHO) compared by Ramel et al. [49]. The conventional fast-food meal was a hamburger meal (hamburger, bacon, and cola drink) and the unconventional fast food was a salmon-burger meal (fiber-rich sourdough rye bread, salad with vinegar, and orange juice). The postprandial increases in glucose and insulin were 44% lower after the unconventional meal, but this effect could be due to the fiber content of this meal.

On the other hand, despite glucose concentrations rise after HFHCM with water and glucose, but not with orange juice, the increase in insulin concentrations was significantly higher with glucose or orange juice compared to water [20]. Accordingly Stookey et al. [23], in a crossover design on 7 adolescents and 10 adults, observed that plasma insulin concentrations were significantly higher after breakfast with orange juice. Furthermore, serum TC and TG did not differ significantly across study days in the adolescents, but TG levels were significantly higher after breakfast with orange juice in adults. On the other hand, Hampton et al. [21] observed a nonsignificant increase in glucose after a meal consisting of vegetable lasagne and cake accompanied with Rabenhorst organic red grape juice and no effect on postprandial TG. The contrasting results on TG of these studies [21, 23] could be due to the different content of fat of the two meals (Table 2). In fact, it is known that the amount of lipid required to cause a significant increase in the levels of TG is of the order of 30–50 g, with low response to 5–15 g [3]. Probably the increase in TG induced by fructose could be appreciated only with low fat meals (LFM).

In this context, 2 consecutive studies were conducted on coronary artery disease (CAD) [50] or healthy subjects [51]. Bae et al. compared the effect of a HFM (803 kcal) which consisted of 110 g rice, 100 g Korean barbecue, 20 g egg, 200 mL milk, 8 g oil, 25 g mayonnaise, and 50 g vegetables (53.4 g fat, 30.7 g protein, and 50 g CHO) and an isocaloric LFM consisting of 312 g rice, 100 g vegetable soup, 200 g vegetables, 190 mL orange juice, 400 g apple, and 50 g kimchi (3 g fat, 15.7 g protein, and 178 g CHO). Authors found decreased postprandial TG and oxidative burst in CAD patients [50], but no effect was observed on TG and malondialdehyde (MDA) in healthy subjects [51]. The different effects could most likely be related to both the healthy status and the different fat content of the meals rather than to the presence of fruit and fruit juice in the LFM.

Only Ghanim et al. [20] investigated the effect of orange juice on the inflammatory markers (Table 2). When a HFHCM (egg-muffin and sausage-muffin sandwiches and 2 hash-brown potatoes) was ingested with water or glucose, there was a significant rise in TLR2 or TLR4 mRNA or protein, as well as of the plasma concentration of endotoxin and oxidative burst. All these effects were inhibited by orange juice (Table 2).

Overall, the results from the studies that have investigated the effect of fruit juice on postprandial stress are scarce and contrasting in drawing any firm conclusion.

## 4. Conclusion

Conflicting results have been reported on the effect of FBD on postprandial stress (Tables 1 and 2). Overall, the results suggest a complex relationship between postprandial dysmetabolism, inflammation, and oxidative stress.

Unfortunately, lipids-challenge has not been standardised and the results cannot be compared very well between studies (Figure 1). Furthermore, the selection of an appropriate control group is a critically important aspect when designing human studies. The purpose of the study dictates the choice of the appropriate placebo. In particular, studies that aim to evaluate the effects of the antioxidants contained in fruit juices should have a placebo identical not only in the total caloric and sugar content but also in the different proportion of glucose and fructose (Figure 1). Only two studies reported the use of a placebo that respects this feature (Table 1). On the other hand, studies that aim to evaluate the effects of FBD as a whole should use water as control, in order to evaluate the effect of both beneficial (antioxidants and fiber) and detrimental (sugars and fructose in particular) components of fruit juice (Figure 1). Also in this case only few studies (Table 2) are available and suggest that orange juice could increase postprandial insulin response. Accordingly, although results from meta-analysis reported that fruit juices did not significantly affect the concentrations of fasting glucose and insulin, they significantly increased the homeostatic model assessment insulin resistance index (HOMA-IR) values [52]. However, while a higher intake of sugar-sweetened fruit juice was significantly associated with a greater risk of T2D, there was no association between the intake of 100% fruit juice and the risk of T2D [53], suggesting that the added sugar was the cause of the increased risk. On the other hand, the high fructose content of the Western-style diet, along with its high fat content, may also be responsible for endotoxemia originating from the gut [54].

Concerning the inflammatory and oxidative stress markers, both markers need further analytical validation and normal ranges should be established in order to draw any firm conclusion. Therefore, caution should be taken in the interpretation of the effect of FBD in postprandial studies and the reviewed results suggest that dietary recommendations should aim to limit rather than increase sugar-sweetened beverages consumption.

## Figures and Tables

**Figure 1:** Difficulty in comparison of postprandial studies and risk of misinterpretation due to control choice. CHO: carbohydrates; FBD: fruit-based drink; HCM: high carbohydrates meal; HFM: high fat meal; M: monocytes, PMN: polymorphonuclear cells; ROS: reactive oxygen species; TG: triglycerides; UA: uric acid.

**Table 1:** Effects of the antioxidants contained in FBD on postprandial stress.

Reference	Subjects (study design)	Control	Treatment	Metabolic markers	Inflammatory and redox markers
Burton-Freeman et al., 2010 [9]	24 OW DL (crossover and parallel)	HFHCM 960 kcal (fat 30.7 g and CHO 134 g) + placebo matched in sugars with HFHCM. 6 weeks placebo matched in sugars, followed by HFHCM + placebo.	HFHCM + strawberry beverage (10 g freeze-dried). 6 weeks strawberry beverage, followed by HFHCM + placebo.	TG ↓ TC ↔ TG, TC ↓	OxLDL ↓ OxLDL ↓,

Edirisinghe et al., 2011 [10]	24 OW DL (crossover)	HFHCM 960 kcal (fat 30.7 g and CHO 134 g) + placebo matched in sugars.	HFHCM + strawberry beverage (10 g freeze-dried).	Glucose ↔ Insulin ↓	IL-6 ↓ IL-1β, TNF-α ↔

Ellis et al., 2011 [11]	24 OW (parallel)	6 weeks placebo matched in sugars, followed by HFHCM 960 kcal (fat 30.7 g and CHO 134 g) + placebo.	6 weeks strawberry beverage (10 g freeze-dried), followed by HFHCM + placebo.	Glucose, insulin ↔	IL-1β, IL-6, TNF-α ↔

Huebbe et al., 2012 [12]	11 OW ATP (crossover)	HFM (cream 200 g and sucrose 75 g) + placebo matched in energy, sucrose, fructose, and glucose.	HFM + FBD (15% Blackcurrant, 9% raspberry, 7% cherry, and 39% red grape).	Glucose, insulin, TG, TC ↔	TNF-α, IL-6 ↑ IL-1*β* ↔ NEAC ↑ oxLDL ↔

Kay and Holub, 2002 [13]	8 (crossover)	HFM 853 kcal (fat 46.7 g and CHO 75.2 g) + placebo matched in CHO and contained 76.4 g of glucose.	HFM + FBD (100 g freeze-dried wild blueberry powder in 500 mL water).	Glucose ↑ TG, TC ↔	NEAC ↑

Mathew et al., 2012 [14]	19 (crossover)	HFM 691 kcal (50 g fat and CHO 56 g) + placebo matched in energy and energy giving nutrients.	HFM + FBD (pomegranate polyphenols 652–948 mg/237 mL). FBD 15 min before the HFM.	Glucose, TG, TC ↔ Glucose, TC ↔ TG ↑	

Mazza et al., 2002 [15]	5 (crossover)	HFM 853 kcal (fat 46.7 g and CHO 75.2 g) + placebo matched in CHO and contained 76.4 g of glucose.	HFM + FBD (100 g freeze-dried wild blueberry powder in 500 mL water).	TG ↔	NEAC ↑

Miglio et al., 2014 [16]	14 OW (crossover)	HFM 1344 kcal (81 g fat and CHO 104 g) + placebo matched in sugars.	HFM + FBD1 (86% of a mix of apple, grape, blueberry, and pomegranate juices and grape skin, grape seed, and green tea extracts). HFM + FBD2 (63% of a mix of pineapple, black currant, and plum juices).		NEAC ↑ isoprostanes ↔ NEAC ↔ isoprostanes ↔

Peluso et al., 2012 [17]	14 OW (crossover)	HFM 1344 kcal (81 g fat and CHO 104 g) + placebo matched in sugars.	HFM + FBD (500 mL; 40% pineapple, 18% blackcurrant, and 5% plum).	Glucose, insulin, TG, TC ↔	TNF-α, IL-6, IL-17 ↓

Peluso et al., 2014 [18]	15 OW (crossover)	HFM 1344 kcal (81 g fat and CHO 104 g) + placebo matched in sugars.	HFM + FBD (500 mL apple juice, red grape juice, pomegranate juice, grape extract from juice, seeds and pomace, raspberry juice, tea extract, ascorbic acid, apple polyphenols, and lemon flavonoids).	Glucose, insulin ↔ TG, TC ↓	TNF-α, IL6 ↓

Snyder et al., 2011 [19]	16 (crossover)	HCM (28 g of Kellogg's Corn Flakes and 118 mL of 2% milk) + placebo matched in energy, sucrose, fructose, glucose, and ascorbic acid.	HCM + navel orange juice (591 mL).		NEAC ↑ dienes ↓

ATP: atherosclerosis prone phenotype; CHO: carbohydrates; DL: dyslipidaemic; FBD: fruit-based drink; HCM: high carbohydrates meal; HFM: high fat meal; HFHCM: high fat and high carbohydrates meal; IL: interleukin; NEAC: nonenzymatic antioxidant capacity; oxLDL: oxidized low density lipoproteins; OW: overweight; TC: total cholesterol; TG: triglycerides; TNF: tumor necrosis factor.

**Table 2:** Studies with water as control.

Reference	Subjects (study design)	Control	Treatment	Metabolic markers	Inflammatory and redox markers
Ghanim et al., 2010 [20]	30 (parallel)	HFM 900 kcal (51 g fat and CHO 81 g) + water *HFM + 300-kcal drink (75 g glucose) *	HFM + orange juice (300 kcal)	Glucose ↓ Insulin ↑ *Glucose ↓* *Insulin ↔ *	Oxidative burst ↓ TLR-2, TLR-4, LPS↓ *Oxidative burst ↓* *TLR-2, TLR-4, LPS↓ *

Hampton et al., 2010 [21]	10 (crossover)	HFM 629 kcal (50% fat and CHO 33.3%) + water	HFM 629 kcal (50% fat and 33.3% CHO) + 122.5 mL Rabenhorst organic red grape juice	Glucose ↔ TG ↔	

Panahi et al., 2013 [22]	29 (crossover)	Pizza and water (fat 32 g, CHO 121.2 g, and sugars 21 g) *Pizza and cola (fat 30.5 g, CHO 166.8 g, and sugars 71.9 g)* *Pizza and diet cola (fat 30.9 g, CHO 116.6 g, and sugars 20.6 g) *	Pizza and orange juice (fat 31.7 g, CHO 178.9 g, and sugars 71.4 g)	Glucose ↑ *Glucose ↔* *Glucose ↑ *	

Stookey et al., 2012 [23]	17 (crossover)	Breakfast with water 1527 KJ (fat 12 g and CHO 55 g)	Breakfast with orange juice 2406 KJ (fat 12 g and CHO 106 g)	Glucose ↔ Insulin ↑ (adolescents) TG ↑ (adults) TC ↔	

CHO: carbohydrates; HFM: high fat meal; LPS: lipopolysaccharide; TC: total cholesterol; TG: triglycerides; TLR: Toll-like receptor.

## Abbreviations

ATP: Atherosclerosis-prone phenotype
CAD: Coronary artery disease
CHO: Carbohydrates
CVD: Cardiovascular disease
DL: Dyslipidaemic
DUR: During
FBD: Fruit-based drink
FRAP: Ferric reducing antioxidant potential
HCM: High carbohydrates meal
HFHCM: High fat and high carbohydrates meal
HFM: High fat meal
HOMA-IR: Homeostatic model assessment insulin resistance index
IBD: Inflammatory bowel disease
IBS: Irritable bowel syndrome
IL: Interleukin
LFM: Low-fat meal
LPS: Lipopolysaccharide
MDA: Malondialdehyde
NAFLD: Nonalcoholic fatty liver disease
NEAC: Nonenzymatic antioxidant capacity
OW: Overweight
oxLDL: Oxidized low density lipoproteins
PRE: Before
ROS: Reactive oxygen species
T2D: Type 2 diabetes
TC: Total cholesterol
TG: Triglycerides
TLR: Toll-like receptor
TNF: Tumor necrosis factor
TRAP: Total radical-trapping antioxidant parameter
UA: Uric acid.
